# Effects of Different Delivery Modes on Pelvic Floor Function in Parturients 6–8 Weeks after Delivery Using Transperineal Four-Dimensional Ultrasound

**DOI:** 10.1155/2022/2334335

**Published:** 2022-05-18

**Authors:** Chao Wang, Qirong Wang, Xuemei Zhao, Xia Wang, Wenji Zhou, Liqing Kang

**Affiliations:** ^1^Graduate School, Tianjin Medical University, Tianjin City 300070, China; ^2^The No. 2 Department of Ultrasound, Binzhou No. 2 People's Hospital, Binzhou, Shandong Province 256800, China; ^3^Maternal and Child Health Planning Service Center of Zhanhua, Binzhou, Shandong Province 256800, China; ^4^Department of Pelvic Floor Disease Rehabilitation and Treatment, Binzhou No. 2 People's Hospital, Binzhou, Shandong Province 256800, China; ^5^Department of Medical Imaging, Cangzhou Central Hospital, Cangzhou Teaching Hospital of Tianjin Medical University, Cangzhou, Hebei Province 061001, China

## Abstract

**Objective:**

To evaluate the effects of different delivery modes on pelvic floor function in parturients 6–8 weeks after delivery using transperineal four-dimensional ultrasound.

**Methods:**

Pelvic floor function 6–8 weeks after delivery in 40 vaginal delivery parturients between November 2018 and December 2020 was assessed by four-dimensional ultrasound, with 40 selective cesarean section delivery parturients as a control group. The imaging results of the two groups were compared.

**Results:**

The levels of clinical indexes such as UVJ-M, *A*_*r*_, *A*_*v*_, *θ*, *D*_*r*_, *D*_*v*_, and ARJ-VDv in the selective cesarean section group were significantly lower than those in the vaginal delivery group 6–8 weeks after delivery (*P* < 0.05). However, no significant difference in CV-VD was observed under Valsalva action and at rest between the two groups (*P* > 0.05). No significant difference in ARJ-VD was found at rest between the two groups (*P* > 0.05). The incidence of pelvic organ prolapse in the selective cesarean section group (40.0%) was significantly lower than that in the vaginal delivery group (62.5%) (*P* < 0.05). No significant difference in the parameters of pelvic diaphragm hiatus at rest was observed between the two groups (*P* > 0.05). The parameters of pelvic diaphragm hiatus under maximum Valsalva action in the vaginal delivery group were significantly higher than those in the selective cesarean section group (*P* < 0.05). Whether the patient was complicated with diabetes had no significant effect on the functional injury of pelvic floor muscle (*P* > 0.05).

**Conclusion:**

The pelvic floor function 6–8 weeks after delivery was significantly more affected in vaginal delivery than in selective cesarean section. Selective cesarean section had certain but limited protective effect on maternal pelvic floor tissue.

## 1. Introduction

With the rapid development of social economy and the continuous improvement of people's living standards, people's health consciousness has been further enhanced, and women of childbearing age pay more and more attention to pregnancy and pelvic floor function [1]. Pelvic floor dysfunction may be caused by pregnancy and childbirth, chronic constipation, and chronic cough, and intense physical exercise may also increase the risk of the disease. The occurrence of pelvic floor dysfunction is also related to age, perimenopausal period, heredity, drugs, lifestyle, and other factors. More than 45% of women were reported to have pelvic floor dysfunction in varying degrees [2, 3]. The progression of female pregnancy will slowly enlarge the uterus and change its position [4]. Especially for women in the third trimester, when the position of the uterus is close to the vertical state, thus, the supporting tissue of the pelvic floor will be under relatively greater pressure [5, 6]. Early detection of pelvic function problems in women is important to the improvement of the therapeutic effect. Transperineal four-dimensional pelvic floor ultrasound has the advantages of easy operation, high accuracy, and less injury; it has also become an important way to detect the function of women's pelvic floor in clinic [7].

The traditional diagnosis is based on anatomical diagnosis of clinical symptoms and mainly uses the POP-*Q* evaluation method. The main examination methods of pelvic floor dysfunction include anorectal manometry, pelvic floor electromyography, perianal, perineal, and intracavitary ultrasound, and defecography. The treatment of pelvic floor dysfunction can be divided into nonoperative treatment and surgical treatment. Nonoperative treatment is the first-line treatment of pelvic organ prolapse (POP). For all patients with organ prolapse, nonoperative treatment should be conducted first. At the same time, it is also suitable for patients who retain reproductive function or cannot tolerate surgical treatment. Surgical treatment can relieve symptoms, increase the strength, endurance, and support of pelvic floor muscles, and prevent the aggravation of prolapse. Patients can also try traditional Chinese medicine and acupuncture. The main purpose of surgical treatment is to relieve symptoms and restore normal anatomical position and organ function. This study is aimed at investigating the effects of different delivery modes on the pelvic floor function of parturients 6–8 weeks after delivery by transperineal four-dimensional pelvic floor ultrasound.

## 2. Materials and Methods

### 2.1. General Information

Eighty parturients who were visited 6–8 weeks after obstetrical delivery in Binzhou No. 2 People's Hospital between November 2018 and December 2020 were divided into the selective cesarean section group (*n* = 40) and vaginal delivery group (*n* = 40) according to the mode of delivery. This study was approved by the Ethics Committee of Binzhou No. 2 People's Hospital, and the informed consents were signed by all patients.

The inclusion criteria were as follows: (1) all parturients were first-born and singleton, (2) no POP occurred before pregnancy, (3) no pelvic floor injury occurred before delivery, (4) no history of chronic cough, (5) no history of constipation, and (6) all parturients participated in the study voluntarily.

The exclusion criteria were as follows: (1) fetal malformations in antenatal examination, (2) complications during pregnancy, (3) pelvic floor injury before delivery, (4) severe medical or surgical diseases, (5) severe mental illness, and (6) parturients cannot participate in the whole study.

### 2.2. Research Methods

A GE-E10 US system was selected as the testing instrument, and the RIC5-9-D endocavity transducer was installed on the instrument. First, let the pregnant woman urinate thoroughly and then check the bladder, keep the bladder in a proper filling state, and ensure that the urine volume was controlled within 50 ml. After the parturient was kept in a supine position, and the lithotomy position was taken, the coupling agent was applied on the vaginal probe, which was covered with a layer of condom, and was placed in the vagina. The uterus, bilateral appendages, and bilateral ovaries were strictly examined. Next, the probe was placed at the position below the external orifice of the urethra, and then the vaginal vestibule position of the two groups of parturients were examined by ultrasound. The indexes of *θ*, *D*_*r*_, *D*_*v*_, *A*_*r*_, *A*_*v*_, CV-VD, UVJ-M, and ARJ-VD of the two groups were examined under Valsava action and at rest.

### 2.3. Research Index

The ultrasonographic results of two groups with different delivery methods were compared, including the posterior angle of vesicourethral angle (*A*_*r*_, *A*_*v*_), the vertical distance of bladder neck to the inferior edge of pubic symphysis (*D*_*r*_, *D*_*v*_), the angle of urethral tilt (*θ*), urethrovesical junction mobility (UVJ-M), the vertical distance of external cervical orifice to the inferior edge of pubic symphysis (CV-VD), the vertical distance between the anorectal junction and the inferior margin of pubic symphysis (ARJ-VD), and pelvic diaphragmatic hiatus parameters. The probability of POP between the two groups was recorded and compared. To ensure the consistency of the inspection results and the accuracy of the data, all tests and data entry were conducted by the same team, and members may not be changed without special reasons in the course of the study.

### 2.4. Statistical Method

The study used the statistical software SPSS25.0 to process the data. Counting data were expressed as (%), and *χ*^2^ test was used to compare the differences of parameters between the two groups. Measurement data were expressed as (^−^*x* ± *s*), and *t*-test was used to compare the differences of parameters between the two groups. Statistical significance was set at *P* < 0.05.

## 3. Results

### 3.1. Demographic Characteristics in the Two Groups

Table 1 summarizes the clinical features of the parturients. All the differences of demographic characteristics between the two groups were not statistically significant (*P* > 0.05).

### 3.2. Characteristics of Pelvic Floor Detected by Transperineal Ultrasound in the Two Groups

The results of perineal ultrasound examination in Table 2 show that the clinical indexes such as UVJ-M, *A*_*r*_, *A*_*v*_, *D*_*r*_, *D*_*s*_, *θ*, and ARJ-VDv in the selective cesarean section group were significantly lower than those in the vaginal delivery group 6–8 weeks after delivery (*P* < 0.05). However, no significant difference in CV-VD was observed between the two groups under Valsalva action and at rest (*P* > 0.05). No significant difference in ARJ-VD in the resting period was found between the two groups with different delivery methods (*P* > 0.05).

### 3.3. Comparison of the Incidence of POP between the Two Groups

The data in Table 3 show that the incidence of POP in the selective cesarean section was 40.0%, which was significantly lower than that of the 62.5% in the vaginal delivery group (*P* < 0.05).

### 3.4. Comparison of Parameters of Pelvic Diaphragmatic Hiatus between the Two Groups at Rest

The data in Table 4 show that the parameters of the pelvic diaphragm hiatus in the resting state between the vaginal group and the selective cesarean section group were statistically insignificant (*P* > 0.05).

### 3.5. Comparison of Parameters of Pelvic Diaphragmatic Hiatus under Maximum Valsalva Action between the Two Groups

The data in Table 5 show that the parameters of the pelvic diaphragm hiatus under the maximum Valsalva action in the vaginal group were significantly higher than those in the selective cesarean section group (*P* < 0.05).

### 3.6. Comparison of Parameters of Pelvic Diaphragmatic Hiatus in Patients with and without Diabetes at Rest and Maximum Valsalva

In this study, 31 pregnant women with diabetes and 49 cases without diabetes were considered. No significant difference was found in left and right diameter, anterior and posterior diameter, and the area of pelvic diaphragmatic hiatus between patients with and without diabetes at rest and under maximum Valsalva action (*P* > 0.05), see Table 6.

## 4. Discussion

The rectum, urethra, fascia, muscles, vagina, and other tissues are located in the pelvic floor tissues. Thus, they can produce a certain load-bearing effect on various tissues and organs in the pelvic cavity. Accordingly, they can effective ensure their anatomical positions. After pregnancy and childbirth, pelvic floor damage may take place in pregnant women, which may causes pelvic organ prolapse, stress urinary incontinence, postpartum urinary incontinence, and other symptoms [8, 9].

### 4.1. Observation and Exploration of Pelvic Floor Anatomy and Function by Transperineal Ultrasound

With the widespread application of ultrasound, CT, and MRI, the anatomical structure of the pelvic floor tissue can be clearly demonstrated [10]. Among them, the ultrasound has the advantages of low cost, no radioactivity, simplicity, high acceptance by patients, and strong reproducibility and is the first choice for the evaluation of pelvic floor dysfunction [11–13]. The pelvic organs, such as the bladder, urethra, pubic bone, bladder neck, and vagina, can be clearly visualized by four-dimensional perineal ultrasound. Under the resting and Valsalva movement state, the pelvic floor function can be evaluated by the mobility parameters of the pelvic organs such as bladder neck, cervix, rectal ampullary, and the angle parameters of urethral tilt angle and urethral rotation angle [14, 15].

### 4.2. Effect of Pregnancy on Pelvic Floor Function

During pregnancy, the uterus will gradually expand and change from the original horizontal position to the longitudinal position in the pelvic and abdominal cavity [16, 17]. Especially for women in the third trimester of pregnancy, the position of the uterus is close to a vertical state, and the pelvic floor supporting tissues will be relatively stressed. With the slowly grow up of uterus, the spine position of pregnant women will bend forward, and the pelvic cavity will be subjected to pressure from the front and lower parts. The dissolution rate of pelvic floor ligament collagen in pregnant women in the third trimester of pregnancy also continues to increase. The ligaments will gradually become loose; although the cervical ring is affected by the combined force of the posterior and inferior, it faces downward as a whole and plays a role in the genital hiatus [18, 19]. When the delivery is completed, the parturient's uterus will no longer continue to receive the force from the front and lower parts, her hormone levels will slowly return to normal, and so will the support force received from the pelvic floor. The cervical ring will also return to its original state [20]. Relevant studies have shown that many physiological changes that occur during pregnancy will be effectively improved within 6–8 weeks in the postpartum period. If the pelvic floor structure and function fails to be repaired in time after delivery, a series of pelvic floor dysfunction diseases may happen, such as genital prolapse, fecal incontinence, and urinary incontinence [21]. Routine pelvic floor function examination should be performed 42 days after delivery, and pelvic floor rehabilitation treatment can be conducted after 42 days of postpartum lochia. The best time for pelvic floor muscle rehabilitation is within 3 months after delivery in order to avoid urinary incontinence, uterine prolapse, and other pelvic floor dysfunction in the future. In addition, pelvic floor rehabilitation treatment can be conducted at any time for menopausal women and elderly patients with pelvic floor dysfunction, such as sneezing leakage, laughter leakage, and chronic pelvic pain. The sooner the treatment start, the better the outcome is.

### 4.3. Structure of the Pelvic Floor Shortly after Delivery Is Affected by Different Modes of Delivery

Hormone secretion in female will change significantly during pregnancy. Thus, the collagen of the pelvic floor ligament will gradually become loosen and dissolved. This condition will reduce the tension of the pelvic floor muscles. In the third trimester of pregnancy, the pelvic floor structure will be compressed by the weight of the uterus, which will affect the pelvic floor structure and function [22, 23]. During the vaginal delivery of the parturient, the vagina will be stretched, which will lead to lacerations of nerves, pelvic floor muscle fibers, birth canal stretch, and perineal lacerations [24]. This study showed that the incidence of POP in the cesarean section group was significantly lower than that in the vaginal delivery group (*P* < 0.05). The different ways that women choose to give birth have different effects on their postpartum pelvic floor structure and function. Compared with cesarean section, vaginal delivery will cause more recent damage to the pelvic floor structure. No matter what kind of delivery was chosen, the mother needs to receive biological treatment or rehabilitation training in time after childbirth to promote the increase in pelvic floor muscle tension and effectively avoid the appearance of pelvic floor dysfunction diseases. In this study, the differences in the parameters of pelvic diaphragm hiatus in patients at rest between the two groups were not statistically insignificant (*P* > 0.05), and the parameters of the pelvic diaphragm hiatus under the maximum Valsalva action in the vaginal group were significantly higher than those in the selective cesarean section group (*P* < 0.05). The pelvic diaphragm hiatus was the weakest area of female pelvic tissue. The uneven force of the female pelvic diaphragm hiatus or the bottom of the pelvic cavity during delivery, especially vaginal delivery, may increase the risk of female pelvic diaphragm hiatus damage, which leads to long-term pelvic floor tissue prolapse and other complications.

### 4.4. Protective Effect of Selective Cesarean Section on Pelvic Floor Function

The results of this study show that the indicators of *A*_*v*_, *A*_*r*_, and UVJ-M in the cesarean section were significantly smaller than those in the vaginal delivery group (*P* < 0.05), indicating that the structure damage and the impairment of pelvic floor function of the vaginal delivery group were more severe than that of the selective cesarean section. Vaginal delivery may damage pelvic floor muscles and fascia tissue, weaken the pelvic organ supporting structure, and change the mobility of pelvic floor and bladder neck position. These changes are important causes of stress urinary incontinence. Cesarean section can effectively prevent the pelvic floor tissue from tearing or dilating, which avoids damage to the urinary tract and effectively protects the early pelvic floor function of the parturient. However, this conclusion has yet to be verified by a large amount of data in the future, and further exploration is needed.

Some studies have shown that the severity of pelvic floor functional disorders is positively correlated with the course of diabetes; that is, the symptoms of pelvic floor functional disorders are more serious when the history of diabetes is longer. Focusing on pelvic floor functional disorders with diabetic symptoms, reducing the severity of pelvic floor dysfunction, and actively controlling the level of blood glucose are important to improve the prognosis of patients and their quality of life. However, in this study, whether diabetes has significant effect on pelvic floor muscle function damage is unclear. This inadequacy may be due to that the included pregnant women have less menstruation, the course of disease is still short, and their blood glucose levels are well controlled. We will include more cases and draw more profound conclusions in future studies.

In summary, the transperineal four-dimensional pelvic floor ultrasonography was performed on women with different delivery methods. Comparing various parameters shows that the pelvic floor function of women with vaginal delivery is significantly more affected than that with cesarean section. Selective cesarean section has a certain protective effect on the pelvic floor tissue of the lying-in woman, but the protective effect is limited.

## Figures and Tables

**Table 1:** Demographic characteristics in the two groups $\left(\bar{x}\pm s\right)$.

Items	Vaginal delivery group (*n* = 40)	Selective cesarean section group (*n* = 40)	*t*	*P*
Age (years)	24.25 ± 1.77	23.62 ± 1.51	1.7	0.093
Height (cm)	163.25 ± 5.82	162.23 ± 5.81	0.789	0.433
Predelivery weight (kg)	62.11 ± 2.71	61.92 ± 2.86	0.309	0.758
Neonatal weight (kg)	3.16 ± 0.83	3.05 ± 0.68	0.648	0.51

**Table 2:** Pelvic floor characteristics detected by transperineal ultrasound in the two groups $\left(\bar{x}\pm s\right)$.

Items	Vaginal delivery group (*n* = 40)	Selective cesarean section group (*n* = 40)	*t*	*P*
*A*_*r*_ (°)	97.69 ± 10.25	92.26 ± 7.52	2.7014	0.009
*A*_*v*_ (°)	145.26 ± 24.72	126.25 ± 22.31	3.6106	0.001
*D*_*r*_ (cm)	24.25 ± 4.26	27.26 ± 3.87	3.3077	0.001
*D*_*v*_ (cm)	9.42 ± 1.25	11.26 ± 4.28	2.6099	0.011
*θ* (°)	46.26 ± 25.26	27.15 ± 21.68	3.6308	0.000
UVJ-M (cm)	22.26 ± 8.28	15.62 ± 7.24	3.8181	0.000
CV-VDr (cm)	26.62 ± 4.26	27.15 ± 6.11	0.4500	0.652
CV-VDv (cm)	14.25 ± 10.06	16.14 ± 10.38	0.8269	0.512
ARJ-VDr (cm)	12.15 ± 3.25	13.26 ± 3.82	1.3997	0.169
ARJ-VDv (cm)	2.13 ± 1.28	3.87 ± 4.28	2.4634	0.000

Abbreviations: *A*_*r*_ and *A*_*v*_: the posterior angle of vesicourethral angle at rest and Valsalva action, respectively; *D*_*r*_ and *D*_*v*_: the vertical distance of bladder neck to the inferior edge of pubic symphysis at rest and Valsalva action, respectively; *θ*: the angle of urethral tilt; UVJ-M: urethrovesical junction mobility; CV-VDr and CV-VDv: the vertical distance of external cervical orifice to the inferior edge of pubic symphysis at rest and Valsalva action, respectively; ARJ-VDr and ARJ-VDv: the vertical distance between the anorectal junction and the inferior margin of pubic symphysis at rest and Valsalva action, respectively.

**Table 3:** Incidence of POP in the two groups.

Items	Vaginal delivery group (*n* = 40)	Selective cesarean section group (*n* = 40)	*χ* ^2^	*P*
Normal	15	24	—	
Abnormal	25	16	—	
Incidence of abnormal	62.50%	40.00%	4.0525	0.044

**Table 4:** Parameters of pelvic diaphragmatic hiatus in two groups of patients at rest $\left(\bar{x}\pm s\right)$.

Items	Vaginal delivery group (*n* = 40)	Selective cesarean section group (*n* = 40)	*t*	*P*
Left and right diameter (cm)	3.59 ± 0.68	3.61 ± 0.72	0.1277	0.911
Anterior and posterior diameter (cm)	4.63 ± 0.87	4.61 ± 0.86	0.1034	0.897
Area (cm^2^)	16.66 ± 4.56	16.56 ± 4.35	0.5135	0.925

**Table 5:** Pelvic diaphragmatic hiatus under maximum Valsalva action in two groups $\left(\bar{x}\pm s\right)$.

Items	Vaginal delivery group (*n* = 40)	Selective cesarean section group (*n* = 40)	*t*	*P*
Left and right diameter (cm)	6.28 ± 0.39	4.48 ± 0.44	19.36	0.000
Anterior and posterior diameter (cm)	7.13 ± 0.57	5.76 ± 0.48	11.64	0.000
Area (cm^2^)	34.76 ± 2.96	20.81 ± 2.18	24.01	0.000

**Table 6:** Comparison of parameters of pelvic diaphragmatic hiatus in patients with and without diabetes at rest and under maximum Valsalva $\left(\bar{x}\pm s\right)$.

Items	Left and right diameter (cm)		Anterior and posterior diameter (cm)		Area (cm^2^)	
	Resting	Valsalva	Resting	Valsalva	Resting	Valsalva
Complicated with diabetes mellitus (*n* = 31)	3.69 ± 0.65	5.4 ± 0.97	4.70 ± 0.78	5.66 ± 0.83	17.35 ± 4.37	28.56 ± 7.14
Without diabetes (*n* = 49)	3.53 ± 0.72	5.37 ± 1.02	4.57 ± 0.90	5.31 ± 0.87	16.14 ± 4.44	27.44 ± 7.73
*t*	1.001	0.142	0.635	1.818	1.192	0.65
*P*	0.32	0.887	0.527	0.073	0.237	0.518

## Data Availability

The analyzed data sets generated during the study are available from the corresponding author on reasonable request.
